# Perioperative left ventricular perforation in incomplete TAVI and completion of the procedure after surgical repair

This article has been retracted.

**DOI:** 10.1186/s13019-022-01925-4

**Published:** 2022-07-07

**Authors:** Giuseppe Nasso, Giuseppe Santarpino, Gaetano Contegiacomo, Giuseppe Balducci, Antongiulio Valenzano, Enrico Moranti, Domenico Scaringi, Giuseppe Speziale, Ignazio Condello

**Affiliations:** 1 Department of Cardiac Surgery, Anthea Hospital, GVM Care and Research, Via Camillo Rosalba 35/37, 70124 Bari, Italy; 2 Department of Cardiac Surgery, Paracelsus Medical University, Nuremberg, Germany; 3 Cardiac Surgery Unit, Department of Experimental and Clinical Medicine, “Magna Graecia” University of Catanzaro, Catanzaro, Italy; 4 Department of Interventional Cardiology, Anthea Hospital, GVM Care and Research, Bari, Italy

**Keywords:** Transcatheter aortic valve implantation, Left ventricular perforation, Cardiopulmonary bypass

## Abstract

**Background:**

The use of transcatheter aortic valve implantation (TAVI) continues to grow worldwide. Despite increased operator experience, evolution of the technique, and deflectable catheters, major complications still occur in ≤ 6% up to 8% of cases. Such major complications have been associated with a 2- to threefold increase in 30-day mortality. Complications specifically involving the aorta, aortic valve annulus, or left ventricle are rare, occurring in only 0.2–1.1% of cases.

**Case presentation:**

We report the case of a 65-year-old female patient with left ventricular lateral wall perforation during incomplete implantation of a TAVI device, and successive percutaneous completion after surgical repair of the lesion under cardiopulmonary bypass. The surgical strategy and the type of surgical treatment depend on the type of perforation. In general, repair of the lesion and aortic valve replacement are performed. Removal of the TAVI prosthesis and excision of the native aortic valve are standard parts of this repair.

**Conclusion:**

Here we propose a safe alternative for the completion of the TAVI approach after surgical repair, which requires close coordination between the members of the heart team (anesthesiologist, perfusionist, cardiologist, nurse and cardiac surgeon).

## Introduction

The use of transcatheter aortic valve implantation (TAVI) continues to grow worldwide [1]. Despite increased operator experience, evolution of the technique, and deflectable catheters, major complications still occur in ≤ 6% up to 8% of cases. Such major complications have been associated with a 2- to threefold increase in 30-day mortality [2]. Complications specifically involving the aorta, aortic valve annulus, or left ventricle are rare, occurring in only 0.2% to 1.1% of cases [3]. In general, repair of the lesion and aortic valve replacement are performed. Removal of the TAVI prosthesis and excision of the native aortic valve are standard parts of this repair.

## Patient information

A 65-year-old female patient undergoing TAVI for severe aortic stenosis. The study was submitted and approved by institutional ethics committee.

## Diagnostic assessment

Echocardiography showed a peak aortic valve velocity of 4.33 m/s, with a peak pressure gradient of 94 mmHg and a mean pressure gradient of 56 mmHg. Left ventricular end-systolic and end-diastolic dimensions were 31.7 mm and 50.0 mm, respectively. The internal diameter of the aortic annulus was 30.7 mm and the aortic sinus diameter was 37.3 mm. The aortic valve area was 0.87 cm^2^. Computed tomography revealed a bicuspid aortic valve of 27.3 mm in diameter according to an aortic annulus perimeter of 85.6 mm, or an aortic valve of 27.4 mm in diameter according to a valve orifice area of 569 mm^2^.

## Therapeutic intervention

A 29 mm Venus-A valve (CoreValve Evolut R, Medtronic, Minneapolis, MN, USA) was implanted. When we used a 20 Fr balloon to dilate the aortic valve, the patient's systolic blood pressure dropped to 70 mmHg in 5 min. Transesophageal echocardiography (TEE) showed a rapidly increasing pericardial effusion. A single-lumen central venous catheter was inserted immediately into the pericardial cavity through the fourth left intercostal space. Five hundred milliliter bright red bloody hemopericardium was drawn out quickly and infused back into the body through the left femoral artery. Blood pressure recovered after the intervention, but pericardial effusion was not improved as monitored by TEE. Simultaneously, the bloody hemopericardium was continuously pumped back into the femoral artery, to prevent any thrombi being infused into the patient, the patient was fully heparinized. Slight perivalvular leak was detected by fluoroscopy and TEE. We observed that the hemopericardium was with bright red blood rather than blue-black color, suggesting a high risk for left ventricular perforation. Indeed, color flow Doppler imaging clearly showed that a bundle of blood from the left ventricle ejected to the pericardial cavity. The patient was anesthetized and intubated, and an urgent full sternotomy (FS) was performed. In order to maintain hemodynamic stability, full anticoagulation with heparin was administered for immediate institution of cardiopulmonary bypass (CPB). Mild hypothermic (34 °C) CPB was established with central cannulation. CPB is performed during simultaneous volume substitution and inotropic support, and active search for a possible problem. This type of resuscitation requires close coordination between the members of the heart team. The correct diagnosis is established by echocardiography, aortography, and/or coronary angiography, or clinically by direct exploration through a median sternotomy. On the left ventricular surface, we found a 1 cm gap, which was 12 mm away from the lateral wall of the left ventricle in proximity of the distal coronary circumflex artery. Blood ejected to the outside of the left ventricle from the gap with every heartbeat (Fig. 1). We performed cardioplegic arrest with cross-clamping. We used two interrupted horizontal mattress sutures with 2-0 Prolene on two felts to close the cleft. CPB and cross-clamp time was 65 min and 23 min, respectively. After protamine administration, the interventional cardiologist completed the TAVI procedure with post-dilation with a 23 Fr balloon and eliminated the residual periprosthetic leak, this was possible as the TAVI valve had been deployed in place, and all that was required was the balloon dilation. Then, the cardiac surgeon inserted the drains and closed the chest.

**Fig. 1:** 1 cm gap on the left ventricular surface

## Follow-up and outcomes

No myocardial infarction, stroke, incision infection, or conduction block occurred post-operatively. The patient was discharged 9 days later.

## Discussion

Owais T. et Al. report that Left ventricular (LV) perforation is one of the rare and most serious complications of transcatheter aortic valve implantation (TAVI). A small LV cavity, a hypercontractile state, a thin muscular wall, and a narrow aorto-mitral angle may be considered potential predictors of the occurrence of LV perforation during TAVI [4]. Nielsen et al. report in their cases TAVI series, that the limitation of the prolonged presence of a stiff guide in LV reduce the risk of perforation [5]. Safe anchoring of the valve should be balanced between using a larger valve to eliminate paravalvular leakage or a smaller valve to prevent possible annulus rupture. Therefore, precise pre-procedural analysis of the device landing zone is mandatory. This includes determination of the size and morphology of all anatomical structures, meticulous identification of possible factors for annular rupture, and correct interpretation of the findings [6]. Although time consuming, this analysis is the most important part of a TAVI procedure, and the heart team can plan a tailored strategy for the individual patient. Furthermore, the characteristics of the guidewires and their appropriate use are also necessary for the success of the procedure. The excessive tension of the preformed guide to the left ventricular apex during prosthesis release was certainly a contributory cause of the event we recorded.

Improvements in devices, procedural techniques, and imaging tools may simplify TAVI and additionally reduce possible complications [7].

The surgical strategy and the type of surgical treatment depend on the type of rupture. In general, repair of the lesion and aortic valve replacement are performed. Removal of the TAVI prosthesis and excision of the native aortic valve are standard parts of this repair [8]. Alternative or bailout treatments, such as placing a second transcatheter valve to seal an annular tear for isolated rupture of the aortic annulus or to close a rupture may not always be successful and are generally not recommended [9]. Here we propose a safe alternative for completion of the TAVI approach after surgical repair, which requires close coordination between the members of the heart team (anesthesiologist, perfusionist, cardiologist, nurse and cardiac surgeon).

## Data Availability

The datasets used and analysed during the current study are available from the corresponding author on reasonable request.

## Abbreviations

TAVI: Transcatheter aortic valve implantation
TEE: Transesophageal echocardiography
CPB: Cardiopulmonary bypass
